This article has been retracted.

# Changes of Multisectoral Collaboration and Service Delivery in Hypertension Prevention and Control before and after the 2009 New Healthcare Reform in China: An Interrupted Time-Series Study

**DOI:** 10.1155/2021/8976625

**Published:** 2021-09-20

**Authors:** Zhifan Zhang, Zhi Hu, Hua Wang, Qingyu Zhou, Chengyue Li, Mo Hao

**Affiliations:** ^1^Research Institute of Health Development Strategies, Fudan University, Shanghai 200032, China; ^2^Collaborative Innovation Center of Social Risks Governance in Health, Fudan University, Shanghai 200032, China; ^3^Anhui Medical University, Hefei, Anhui 230032, China; ^4^Jiangsu Preventive Medicine Association, Nanjing, Jiangsu 210009, China

## Abstract

**Objectives:**

There is a need to assess the 2009 new healthcare reform in China on hypertension prevention. It helps to control from the perspectives of multisectoral participation, government responsibility assignment, performance assessment, and service delivery.

**Design:**

Interrupted time-series study. *Setting*. 31 provinces in mainland China. *Primary and Secondary Outcome Measures.* Based on the content analysis of publicly available policy documents from 31 provinces regarding hypertension prevention and control, we analyzed the changes brought by the 2009 new healthcare reform through four quantitative indicators, including multisector participation (MP), main department responsibility coverage (MDRC), primary department assessment indicator coverage (MDAIC), and service type coverage (STC). We compared the changing trends of four indicators before and after 2009.

**Results:**

Nationally, MP, MDRC, and STC grew rapidly and increased to 88.9%, 96.4%, and 77.8%, respectively, in 2017, higher than MDAIC (36.9%). This growth was accelerated by the new healthcare reform, with the highest acceleration in MP (*β*3 = 6.345, *p* < 0.001), followed by MDRC (*β*3 = 3.829, *p* < 0.01), STC (*β*3 = 3.799, *p* < 0.001), and MDAIC (*β*3 = 3.585, *p* < 0.001). The MP and MDRC trend changes were higher in the central and western regions than in the east after the reform.

**Conclusions:**

Our research showed that the new healthcare reform had a positive effect in promoting multisectoral participation in preventing and controlling hypertension in China, improving the responsibility mechanism, and expanding the types of services provided. The government should lead the coordination and implementation of multidepartmental responsibilities and mobilize nonhealth departments to continuously participate in the prevention and control of chronic diseases by improving incentive and evaluation mechanisms.

## 1. Introduction

Hypertension is a serious threat to the health of Chinese residents with a prevalence of 23.2% in adults, 41.3% being in the prehypertension stage [1]. This prevalence has increased since the 1990s [2, 3]. Compared to the beginning of the century, hypertension awareness, treatment, and control rates among Chinese residents have increased [1, 4] but are still low [2, 5–8]. Compared to developed countries, there is a gap in hypertension prevention and control effectiveness in China [1, 4]. Many cases of hypertension have not been detected and treated timeously [7, 9], causing a potential for hypertension to burden the Chinese health system.

Since 2005, primary healthcare institutions in 23 provinces across China have gradually carried out standardized management of hypertension [10]. The implementation of the new healthcare reform in 2009 made hypertension prevention and controlled a national government-led project. The reform contained two highlights: first, the government was determined to build a health service network using primary healthcare institutions as the mainstay for providing chronic disease management and rehabilitation services. Second, primary healthcare institutions included hypertension management in the scope of essential public health services provided free of charge [11]. Services included free annual blood pressure measurement for residents aged above 35 and follow-up services for patients with hypertension at least four times a year.

After the reform, provincial governments started attaching importance to hypertension prevention and control. Provinces actively carried out evaluations of the effectiveness of hypertension interventions [10], and patients' blood pressure control rates increased significantly [12, 13]. By the end of 2014, over 86 million hypertension patients were included in standardized hypertension management in primary healthcare institutions [14]. The 2012 “China Chronic Disease Prevention and Control Plan” further indicated that multiple departments should jointly take responsibility for preventing and controlling hypertension.

Chinese researchers have popularised research comparing Chinese healthcare pre- and postreform. Regarding population-based hypertension management, the proportion of patients aware of their conditions, receiving treatment and regular monitoring, and with hypertension under effective control have increased since 2009 [15–17]. The reform narrowed the inequity of hypertension management across regions, with the highest improvement found in undeveloped provinces [16]. Regarding changes in resource allocation and service utilization of primary healthcare institutions and hospitals caused by the reform, there has been a significant increase in the number of hospitals and primary healthcare institutions, and also a noticeable growth in government fiscal subsidies, medical facilities, and the number of health practitioners in county hospitals and community health centers nationwide [18–22]. It is clear that the reform has made significant progress in population health management and health sector resource investment. This could not be achieved without the joint efforts of multiple departments. However, it is unknown how the reform affected the multisectoral participation and construction of government accountability mechanisms which is currently of great concern to the WHO [23, 24]. Thus, our research attempted to fill this gap and specify the changes brought by the reform on hypertension prevention and control from the aspects of multisectoral collaboration and service delivery.

## 2. Method

### 2.1. Study Design

First, we used an interrupted time-series analysis with a breakpoint to assess the changes before and after 2009 on hypertension prevention and control. In 2009, the State Council released *Opinions on Deepening the Reform of the Medical and Health Care System* and *Notice on Issuing the Plan on Recent Priorities in Carrying out the Reform of Health Care System (2009–2011)* in which implementing standardized management of hypertension patients and improving prevention and treatment services were the main contents [11, 25]. To test the reform's impact, we took 31 provinces in mainland China as the research settings. We used content analysis to compare trend changes in multisectoral participation, responsibility assignment, assessment mechanism, and service provision in hypertension prevention and control before (2000–2008) and after 2009 (2009–2017). We assumed that the reform could accelerate the progress of hypertension prevention and control from the aspects of multisectoral participation, responsibility assignment, assessment mechanism, and service provision.

### 2.2. Evaluation Framework and Indicators

We chose Donabedian's model as the theoretical framework to guide the evaluation. Donabedian model, which contains structure, process, outcome, was widely regarded as the basic framework for public health system performance measurement [26–28]. The model was widely used in the evaluation of various links of public health service, such as the evaluation of treatment outcomes (outcome), quality of service provision (outcome), and general practitioners training program (process). [29–32].

As mentioned in the introduction, many studies chose population-level or community-level indicators, such as patient management rate, number of practitioners, and fiscal subsidy, to analyze the reform impact. Our study was based on the macroperspective of health governance. It analyzed the changes in multisectoral cooperation (structure) and service delivery (process) in hypertension prevention and control before and after the reform. We designed four indicators to reflect multisectoral participation and service delivery as shown in Table 1. A 30-member expert panel composed of policymakers, public health practitioners, or researchers reached a consensus on the selection and design of indicators.

In structure, multisectoral participation is an integral part of many public health efforts to deal with chronic diseases such as hypertension. It is also the basis for organizations to obtain valuable human and financial resources [33]. So the indicator multisector participation (MP) was designed to reflect the scope of the departments involved. The higher the indicator, the more departments are involved.

On this basis, the central departments play a vital role in service delivery and health resources allocation. Meanwhile, clear responsibility assignment is necessary for the management of relationships between main departments [34]. The indicator primary department responsibility coverage (MDRC) was designed to reflect how many had clear responsibility assignments. For example, the hospital should measure blood pressure for first-visit patients over the age of 35, clearly describing hospital responsibilities.

In the process, comprehensiveness and accountability are key characteristics of good service delivery, which is also a vital component of the health system [34]. The indicator service type coverage (STC) was designed to reflect whether the types of service coverage are comprehensive; in other words, how many types of services were provided.

Besides, setting assessment indicators for central departments is essential to measuring the actual supply of services [34]. The main department assessment indicator coverage (MDAIC) reflected how many main departments were set with evaluation indicators. For example, the management rate of hypertension patients in primary healthcare institutions needs to be greater than or equal to 60% to set evaluation indicators for primary healthcare institutions to measure performance.

According to the WHO's and China's policy documents [35, 36], we believe that at least 22 stakeholders should be involved in the prevention and control of hypertension, including the provincial government, four actors in the health sector (health commission/public health agencies/hospitals/primary healthcare institutions). Four vital supporting departments (development and reform commission/healthcare security administration/finance bureau/human resources and social security bureau), 12 other supporting departments (education commission/civil affairs bureau/agriculture and rural affairs bureau/transportation commission/drug regulation administration/sports administration/housing bureau/environment bureau/radio and television administration/information and industry technology bureau/commerce commission/work safety administration), and nongovernment organizations (colleges, universities, foundations, etc.). Therefore, we defined the provincial government, four actors in the health sector, and four critical supporting departments as the paramount hypertension prevention and control departments. Additionally, we divided hypertension prevention and control services into eight categories: health education, baseline survey, risk factor surveillance, risk factor interventions, high-risk population screening, related disease surveillance, new care report, and patient management (Appendix 1 in Supplementary Materials).

## 3. Data Collection

### 3.1. Policy Documents Inclusion and Exclusion

In the first stage, a detailed and extensive review was performed to identify relevant policy documents directly or indirectly addressing hypertension prevention and control from 31 provincial governments' official websites in mainland China; these included policy release columns on the websites of provincial governments, health commissions, development and reform commissions, CDCs, etc. Then, supplementary searches for terms, such as “hypertension,” “chronic disease” combined with “regulation,” “plan,” “guideline,” “standard,” and “decision,” were carried out on the government websites. The inclusion criteria were (1) publicly available and administratively valid government documents, including laws or regulations, strategic plans, guidelines, decisions, and standards; (2) released before the end of 2017; and (3) only provincial-level policies. The exclusion criteria were (1) nonbinding documents or documents without administrative validity, including news and reports and (2) not having specific publication dates. A total of 742 documents from 31 provinces were included (Appendix 2 in Supplementary Materials).

### 3.2. Information Coding

We clarified each document's year of publication and extracted and coded the information required by the four quantitative indicators in the documents (Appendix 3 in Supplementary Materials). Taking multisector participation (MP) as an example, we established whether the 22 department categories were mentioned in the documents. For example, if a document mentioned that the prevention and control of hypertension are organized and implemented by the CDC, the CDC as a public health agency was considered involved in the prevention and control of hypertension. Thus we coded public health agency as 1. By determining whether each department was mentioned in the documents, the number of departments mentioned was accumulated to obtain the numerator, divided by 22 (number of departments) to obtain the MP value. We recorded the original description in the documents so that coding can be checked and substantiated. Excel 2010 was used to organize the data and calculate each indicator. Documents were coded according to the coding template, and two team members reviewed the data independently.

### 3.3. Data Analysis

We used the interrupted time-series (ITS) model to evaluate the indicators levels and trends pre- and postreform with Newey–West corrected SEs (which account for autocorrelation) [37, 38]. ITS models with interruption points were formulated to detect the effect on indicators yearly as follows:

(1) $$\begin{array}{c} Y_{t}=\beta_{0}+\beta_{1}\times {\text{time}}_{t}+\beta_{2}\times \text{new healthcare reform }2009+\beta_{3}\times \text{time after }{\text{reform}}_{t}+\varepsilon_{t}. \end{array}$$

We used *β*_0_ to estimate the baseline level of each indicator; *β*_1_ estimated the baseline trend of each indicator prereform; *β*_2_ estimated the change in level postreform; *β*_3_ estimated the change in trend postreform; *ε*_*t*_ is an estimate of the random error at time _*t*_. We used the Cumby–Huizinga test for the autocorrelation of each indicator. If autocorrelation is presented at higher lag orders (up to the six lags tested), we revised the lag orders in the model to account for this. The value of the MDAIC in the west and central regions was 0 for 2000–2008. We used corresponding data from 2009–2017 to perform regression prediction on the value of 2000–2008 to fit the ITS Analysis [39].

Our research data covered all 31 provinces in mainland China, and we divided the 31 provinces into three geographical regions: east (include 11 provinces), central (including 8 provinces), and west (including 12 provinces) according to the national standard [40]. We analyzed the changes before and after the reform on four quantitative indicators across regions. All analyses were completed using Stata V.15.0, and *p* value <0.05 was considered statistically significant.

### 3.4. Patient and Public Involvement

Patients or the public WERE NOT involved in our research's design, conduct, reporting, or dissemination plans.

## 4. Results

### 4.1. General Descriptions of Four Indicators

The starting points of four indicators in 2000 were all below 10% nationally with a continuous upward trend thereafter. MP, MDRC, and STC multiplied and increased to 88.9%, 96.4% and 77.8%, respectively, in 2017, higher than MDAIC (36.9%) in the same year (Table 2). Regionally, the 2000 baseline levels of the MP and MDRC in the east were better than in the central and western regions. However, by 2017, the gap had diminished. The baseline level of the MDAIC was 0% in all three regions in 2000. By 2017, the east (44.4%) was better than that of the central (36.1%) and the west (30.6%). Although the western region had a higher baseline level of STC in 2000, the eastern region still outperformed the central and western regions in 2017.

### 4.2. Influence of Reform on Structure Indicators

In terms of the national average, MP grew slowly between 2000 and 2008 (*β*1 = 1.117, *p* < 0.001). After the reform, MP increased suddenly (*β*2 = 20.203, *p* < 0.01) and somewhat faster between 2009 and 2017 (*β*3 = 6.345, *p* < 0.001) (Table 3 and Figure 1). Regionally, before 2009, the growth trend of MP in the eastern region (*β*1 = 1.278, *p* < 0.001) was higher than in the central (*β*1 = 1.127, *p* < 0.01) and western regions (*β*1 = 0.957, *p* < 0.001). From 2009 to 2017, the growth trend of MP accelerated among all regions, and the most rapid increase occurred in the west (*β*3 = 7.547, *p* < 0.001).

MDRC was similar to MP in baseline level and trend. However, nationally, MDRC increased suddenly in 2009 (*β*2 = 32.188, *p* < 0.001) and faster (*β*3 = 3.829, *p* < 0.01) than in the baseline period. Regionally, the west and the central regions showed higher level and trend change relative to the east.

### 4.3. Influence of Reform on Process Indicators

The growth of nationwide MDAIC accelerated postreform (*β*3 = 3.585, *p* < 0.001) (Table 4 and Figure 1). However, regionally, only the east showed a significant level (*β*2 = 5.044, *p* < 0.05) and trend change (*β*3 = 3.905, *p* < 0.001) postreform. Thus, the MDAIC in the western and central regions only experienced a sudden increase in 2009.

In terms of the national average, STC grew slowly during 2000–2008 (*β*1 = 1.739, <0.001), postreform, STC increased suddenly (*β*2 = 14.951, *p* < 0.01) and faster during 2009–2017 (*β*3 = 3.799, *p* < 0.001) (Table 4 and Figure 1). Regionally, the three regions had a slight upward trend from 2000–2008, but the eastern (*β*1 = 2.172, *p* < 0.001) and central regions (*β*1 = 2.917, *p* < 0.001) grew faster than the western (*β*1 = 0.555, *p* < 0.01). In 2009, the reform had a sudden increase in STC in all three regions, but the change was most obvious in the eastern region (*β*2 = 18.840, *p* < 0.01). Opposite to the baseline trend, the growth of STC in the west accelerated the fastest (*β*3 = 5.988, *p* < 0.0001) among the regions.

## 5. Discussion

To our knowledge, this study was the first attempt to use quantitative analysis to evaluate the changes brought by the reform on hypertension prevention and control in China from the perspective of multisectoral participation, responsibility assignment, performance assessment, and service provision. As a result, the reform accelerated the improvement of the above four aspects at the national level.

The reform had the most obvious influence on multisector participation and responsibility assignment, indicating that the government has realized the importance of multisectoral collaboration in hypertension prevention and control after 2009, providing a primary platform for routine coordination between departments. Several factors have contributed to this phenomenon. Firstly, postreform, the government began to explore a chronic disease prevention and control model centered on a government-led, multisectoral participation, whole-of-society approach. The prevention and treatment of hypertension were a core task of this exploration and have been a priority for chronic disease prevention and control in China. The most prominent action was that the National Demonstration Area for comprehensive prevention and control of noncommunicable disease (NDA) had been launched in all provinces since 2010, a project with transfer payments from the national government [41]. The establishment of the NDAs built a multisectoral coordination platform for the prevention and control of hypertension led by the health department. Early detection and management of hypertension was the focus task in the NDAs, and assessment indicators were set to ensure the health departments implemented the tasks effectively. Secondly, in 2012, the Ministry of Health and 15 other departments issued China's first chronic disease prevention and control plan [42]. The plan clarified that development and reform, education, finance, human resources, and social security, and sports departments should participate in chronic disease prevention and control. The national plan provided a policy-support environment for preventing and controlling hypertension across the country and a policy guarantee for multisectoral cooperation. Following the plan's introduction, in 2013, 15 provinces successively released chronic disease prevention and control plans jointly formulated by multiple departments [43].

Some previous studies have also reached similar conclusions after reform cooperation among multiple departments had been strengthened. Health departments in various provinces established transdepartmental cooperation for the prevention and control of chronic diseases and clarified the scope of the responsibilities of each department [44, 45]. Further, the number of provincial CDCs cooperating with departments within the health sector (hospitals and primary health institutions) and the number of provincial CDCs cooperating with departments outside the health sector (education and sports departments) for chronic disease prevention and control both increased after 2009 [46]. Since hypertension prevention and control require the participation and clear responsibility assignment of multiple government departments, our study provides evidence on whether the reform promotes establishing a multisectoral cooperation mechanism for hypertension management from a broader perspective.

The study found that the comprehensiveness of service provision has also improved rapidly after 2009. Other studies have reached similar conclusions. After 2009 there was an increase in patient identification, health records establishment, medication treatment, and health education among hypertension patients [18, 47]. Besides, the standardization of services provided by primary healthcare providers has been strengthened [17]. The main reason was that the former Ministry of Health issued a national regulatory document to standardize hypertension patients' early detection and management [48]. After the policy was released, hospitals and primary healthcare institutions cooperated in providing services such as health education, baseline surveys, screening, etc. The provincial CDC played a coordinating and supervising role to ensure the effectiveness of service delivery.

Our results also showed that there is still room for improvement in the design of departments' performance assessment mechanisms. For example, many provincial governments only included the standardized management rate of hypertension patients in the annual performance assessment of primary healthcare institutions and health departments [49, 50]. This approach failed to restrict other departments outside the health sector directly. This indicates that the main responsibilities for hypertension prevention and control are still within the health sector, as other departments have not been actively mobilized to participate and effectively implement hypertension-related policies. Researchers have pointed out that the health sector in China is in a relatively weak position among all government departments and does not have effective administrative power when coordinating multisector participation for the prevention and control of chronic diseases [51]. Further, nonhealth departments do not incorporate chronic disease prevention and control into their work plans or arrangements; thus, enthusiasm for participating in chronic disease prevention and control and implementation efficiency is low [41, 52].

Regionally, the growth trends of all indicators in the eastern region before 2009 were higher than the national average, suggesting that hypertension prevention and control in the east started earlier. Due to the advantages of economic development, the prevalence and growth rate of hypertension in eastern provinces were comparatively higher [53]. This phenomenon forced the eastern region to establish a service provision system earlier to meet the population's health needs. Some provinces in the eastern region explored hypertension management at the primary care level. Beijing and Shanghai carried out community intervention trials for hypertension management before 2000 [50] and subsequently evaluated the effectiveness of the project [52, 54]. The Disease Control Bureau of the former Ministry of Health selected 23 provinces for pilot projects in 2005 to explore the model and experience of standardized management of hypertension in the community, covering most provinces in the eastern region [10].

In comparison, MP and MDRC in the central and western regions after 2009 were higher than in the east. The backward development of chronic disease management in those regions was mainly due to the government's early lack of health investment. Weak medical infrastructure has hindered the prevention and control of chronic disease in these two regions. Until 2009, the national government invested significant funding to establish regional hospitals and community healthcare centers in less-developed rural and western regions [55] and the central and western regions to promote a chronic disease management mechanism further.

Our findings have some policy implications for strengthening hypertension prevention and control measures. First, based on the establishment of the NDAs, an authoritative coordinator, such as the health department or the provincial government, should be appointed to coordinate routine affairs, and a multisectoral cooperation mechanism should be formed among multiple departments. Second, China needs to formulate laws and regulations for preventing and controlling hypertension and other chronic diseases, and the responsibilities of nonhealth departments need to be clarified or strongly restricted. Besides, the task of chronic disease prevention and control should be included in the work plan of the relevant nonhealth departments. Assessment indicators for the work of these nonhealth departments need to be set to enhance their enthusiasm. Third, the national government's health investment should continue to focus on the central and western regions. Although the central and western regions grew rapidly after 2009, there was still a gap in the eastern regions. In addition to medical infrastructure, the national investment in health should also focus on how to help the central and western regions attract and retain high-quality health human resources to improve the overall management of chronic diseases in those regions.

There are several limitations to this study. First, the findings mainly reflected the overall developmental performance of China and the eastern, central, and western regions, while the analysis of a specific province is not thorough enough. Future studies research could focus on a single well-performing province to clarify its unique development advantages. However, we provided a reference to the general condition of the whole country for further in-depth research. Second, we only designed and analyzed the structure and process indicators according to Donabedian's model. We did not analyze the changing trend of the outcome indicators and their relationship to the other indicators. We could collect health outcome indicators such as hypertension prevalence and management rate and adopt mixed methods for further analysis. Third, in our analysis, changes in trends of the four indicators may be affected by factors, such as political and economic environment, allocation of health human and finance resources, the prevalence of hypertension, etc., nationwide or in different regions. In a further study, we will explore the association between these factors and the four indicators.

## 6. Conclusions

Our quantitative study was the first to clarify the positive effect of the health reform on multisectoral participation and responsibility division in hypertension prevention and control. The findings indicate that there is still room for improvement in developing a government-based performance assessment mechanism. Regionally, the central and western regions have made progress in hypertension management following the reform. The government should act as the primary leader to coordinate and implement multidepartmental responsibilities and further mobilize nonhealth departments to continuously participate in the prevention and control of chronic diseases by improving incentive and evaluation mechanisms.

## Figures and Tables

**Figure 1:** Trend changes of 4 indicators before and after 2009 new healthcare reform, 2000–2017.

**Table 1:** Definition of the four indicators.

Dimension	Indicator name	Definition
Structure	Multisector participation (MP) (%)	The percentage of departments/organizations that actually participated from the 22 departments that should be included in hypertension prevention and control

Process	Main department responsibility coverage (MDRC) (%)	The percentage of departments/organizations with responsibilities assigned from among the nine main departments that should be included in hypertension prevention and control
	Main department assessment indicator coverage (MDAIC) (%)	The percentage of departments/organizations with assessment indicators from among the nine main departments that should be included in hypertension prevention and control
	Service type coverage (STC) (%)	The percentage of services provided among the eight service types that should be included in hypertension prevention and control

**Table 2:** Comparison of indicators by region from 2000 to 2017.

	Nationwide		East		West		Central	
	2000	2017	2000	2017	2000	2017	2000	2017
MP (%)	3.2	88.9	9.1	89.3	0.0	87.3	0.0	90.8
MDRC (%)	5.7	96.4	16.2	98.0	0.0	97.2	0.0	93.1
MDAIC (%)	0.0	36.9	0.0	44.4	0.0	30.6	0.0	36.1
STC (%)	3.9	77.8	3.0	81.8	7.4	75.0	0.0	76.4

MP, multisector participation; MDRC, main department responsibility coverage; MDAIC, main department assessment indicator coverage; STC, service type coverage.

**Table 3:** Results of interrupted time-series analysis of the changes before and after 2009 on structure indicators.

	Multisector participation (MP) (%)				Main department responsibility coverage (MDRC) (%)			
	Nationwide	East	West	Central	Nationwide	East	West	Central
Baseline level (*β*0)	1.286	7.02^*∗∗∗*^	−1.582	−2.284	2.712	12.906^*∗∗∗*^	−3.415	−2.098
Baseline trend (*β* 1)	1.117^*∗∗∗*^	1.278^*∗∗∗*^	0.957^*∗∗∗*^	1.127^*∗∗*^	2.170^*∗∗∗*^	2.946^*∗∗∗*^	2.037^*∗∗∗*^	1.296^*∗∗∗*^
New healthcare reform 2009 level change (*β*2)	20.203^*∗∗*^	24.906^*∗∗∗*^	16.97^*∗*^	18.644^*∗∗*^	32.188^*∗∗∗*^	25.367^*∗∗*^	37.883^*∗∗*^	33.058^*∗∗∗*^
New healthcare reform 2009 trend change (*β*3)	6.345^*∗∗∗*^	4.791^*∗∗∗*^	7.547^*∗∗∗*^	6.682^*∗∗∗*^	3.829^*∗∗*^	1.818^*∗*^	4.799^*∗*^	5.140^*∗∗∗*^

^*∗*^*p* ≤ 0.05; ^*∗∗*^*p* ≤ 0.01; ^*∗∗∗*^*p* ≤ 0.001.

**Table 4:** Results of interrupted time-series analysis of the changes before and after 2009 on process indicators.

	Main department assessment indicator coverage (MDAIC) (%)				Service type coverage (STC) (%)			
	Nationwide	East	West	Central	Nationwide	East	West	Central
Baseline level (*β*0)	−0.302	−0.853	0.429^*∗∗∗*^	0.077	1.326	−0.045	6.32^*∗∗∗*^	−4.259
Baseline trend (*β*1)	0.185^*∗∗*^	0.522^*∗∗*^	−0.101	−0.010	1.739^*∗∗∗*^	2.172^*∗∗∗*^	0.555^*∗∗*^	2.917^*∗∗∗*^
New healthcare reform 2009 level change (*β*2)	3.029^*∗∗*^	5.044^*∗*^	2.612^*∗∗∗*^	3.809^*∗∗∗*^	14.951^*∗∗*^	18.840^*∗∗*^	15.395^*∗*^	8.964^*∗∗*^
New healthcare reform 2009 trend change (*β*3)	3.585^*∗∗∗*^	3.905^*∗∗∗*^	−0.691	−0.180	3.799^*∗∗∗*^	2.779^*∗∗*^	5.988^*∗∗∗*^	1.922^*∗∗*^

^*∗*^*p* ≤ 0.05; ^*∗∗*^*p* ≤ 0.01; ^*∗∗∗*^*p* ≤ 0.001.

## Data Availability

No data are available.

## Supplementary Materials

Supplementary Materials Supplementary material for the study contains Appendices 1, 2, and 3. Appendix 1 defines eight categories of hypertension prevention and control services in the study, which include health education, baseline survey, risk factor surveillance, risk factor interventions, high-risk population screening, related disease surveillance, new care report, and patient management. Appendix 2 provides a flowchart for the selection of policy documents in the study, which includes four stages of identification, screening, eligibility, and inclusion. Appendix 3 provides the coding instruction of four indicators in the study.
